The article "Investigating the Molecular Mechanism of Quercetin Protecting against Podocyte Injury to Attenuate Diabetic Nephropathy through Network Pharmacology, MicroarrayData Analysis, and Molecular Docking" was published in 2022. Journal: Evid Based Complement Alternat Med.

# Investigating the Molecular Mechanism of Quercetin Protecting against Podocyte Injury to Attenuate Diabetic Nephropathy through Network Pharmacology, MicroarrayData Analysis, and Molecular Docking

**DOI:** 10.1155/2022/7291434

**Published:** 2022-05-16

**Authors:** Xiaoqin Ma, Chenxia Hao, Meixiang Yu, Zhaokang Zhang, Jingjing Huang, Wanhua Yang

**Affiliations:** ^1^Department of Pharmacy, Ruijin Hospital, Shanghai Jiaotong University School of Medicine, Shanghai 200025, China; ^2^Department of Pharmacy, Xi'an Children's Hospital, Xi'an, China; ^3^Department of Pharmacy, Shanghai Children's Medical Center, Shanghai Jiao Tong University School of Medicine, Shanghai, China

## Abstract

Quercetin (QUE), a health supplement, can improve renal function in diabetic nephropathy (DN) rats by ameliorating podocyte injury. Its clinical trial for renal insufficiency in advanced diabetes (NCT02848131) is currently underway. This study aimed to investigate the mechanism of QUE protecting against podocyte injury to attenuate DN through network pharmacology, microarray data analysis, and molecular docking. QUE-associated targets, genes related to both DN, and podocyte injury were obtained from different comprehensive databases and were intersected and analyzed to obtain mapping targets. Candidate targets were identified by constructing network of protein-protein interaction (PPI) of mapping targets and ranked to obtain key targets. The major pathways were obtained from Kyoto Encyclopedia of Genes and Genomes (KEGG) and Gene Ontology (GO) term enrichment analysis of candidate targets via ClueGO plug-in and R project software, respectively. Potential receptor-ligand interactions between QUE and key targets were evaluated via Autodocktools-1.5.6. 41. Candidate targets, of which three key targets (TNF, VEGFA, and AKT1), and the major AGE-RAGE signaling pathway in diabetic complications were ascertained and associated with QUE against podocyte injury in DN. Molecular docking models showed that QUE could closely bind to the key targets. This study revealed that QUE could protect against podocyte injury in DN through the following mechanisms: downregulating inflammatory cytokine of TNF, reducing VEGF-induced vascular permeability, inhibiting apoptosis by stimulating AKT1 phosphorylation, and suppressing the AGE-induced oxidative stress via the AGE-RAGE signaling pathway.

## 1. Introduction

Podocyte injury is a critical event resulting in the eventual podocyte loss in the development and progression of diabetic nephropathy (DN), accounting for 40–45% of patients with diabetes mellitus [1–3]. Moreover, podocytes and podocyte-specific proteins are potential urinary markers to detect the early diagnosis of DN, and low podocyte density, correlating directly with the magnitude of proteinuria, is a strongest predictor for progression of DN [4]. Furthermore, podocyte injury results in permanent alterations in the glomerular filtration barrier in DN [5, 6]. Podocytes are core cells of the glomerular filtration barrier and terminally differentiated parietal epithelial cells with a very limited proliferation ability [7].

Recently, podocyte injury has been regarded as a novel early mechanism involved in DN [8]. In the progress of DN, hyperglycemia (HG) induces the excessive accumulation of advanced glycation end products (AGEs) with reactive oxygen species (ROS), initiating podocyte injury accompanied with proteinuria and ultimately accelerating the development of DN [9, 10]. Podocytes are also targets of AGEs in diabetes by increasing AGE receptor (RAGE) expression [11]. The activated AGE-RAGE signaling pathway (AGEs binding to RAGE) increasing expressions of proinflammatory cytokine and oxidative stress is closely associated with podocyte injury and has been confirmed exactly one of the mechanisms of DN occurrence [12, 13]. However, the alleviation of podocyte injury in DN is mainly to control HG or proteinuria for the management of renal damage [3, 14], but lacks targeted agents. So, drugs targeting podocyte injury are urgently needed to treat DN and will be one of the most promising field of inquiry [13].

Quercetin (3,3′,4′,5,7-pentahydroxyflavone, QUE) belongs to natural flavonoids that are commonly defined as dietary antioxidants [15]. It has significant therapeutic effects on DN by reducing proteinuria which is a typical clinical manifestation mostly resulted from the podocyte injury [16, 17]. Moreover, it can reduce the oxidative stress, inflammatory responses and apoptosis involved in the progression of DN [18, 19]. Many clinical trials of QUE, including clinical research for renal insufficiency in advanced diabetes (clinicaltrials.gov ID NCT02848131) are currently underway (https://www.clinicaltrials.gov/) [20, 21]. In vitro experiments have confirmed that QUE reverses diabetes-induced podocyte injury by increasing the expression level of nephron and podocin in podocytes [20, 22, 23].

QUE is a phytochemical contained in many Chinese herbs such as *Astragalus membranaceus* (ASM) and *Salvia miltiorrhiza bunge* (SMB). ASM has been reported to have protective effects on podocyte injury and SMB can ameliorate diabetic vascular injury in streptozotocin-induced diabetic rats [24, 25]. However, the molecular mechanism of protects against podocyte injury in DN is lacking. Fortunately, network pharmacology can decipher the mechanism of drugs action with a holistic perspective, which breaks through the “one drug, one target” in the traditional drug discovery model and realizes the synergy of multiple targets [26]. Hence, this study aimed to investigate the mechanism of QUE protecting against podocyte injury to treat DN through network pharmacology [26], microarray data analysis, and molecular docking.

## 2. Materials and Methods

The flowchart of this study design about the network pharmacology method used to clarify the key targets and the major pathway of QUE protecting against podocyte injury is shown in Figure 1, including six parts: searching QUE-associated targets, screening genes related to DN and podocyte injury, retrieving of mapping target interaction proteins, constructing protein-protein interaction (PPI) network, enrichment analysis, and molecular docking.

### 2.1. Searching QUE-Associated Targets

Targets of QUE were searched from the following three databases with the keyword “quercetin.” One is the Traditional Chinese Medicine Systems Pharmacology database [27] (TCMSP, https://lsp.nwu.edu.cn/) which focuses on the exploration of the targets from the HIT database, SysDT model, and targets validated by experiments [27]. Another is the SwissTargetPrediction database [28] (https://www.swisstargetprediction.ch) which estimates the most probable targets of QUE in view of 2D and 3D similarity between QUE and known activities in this database [29]. The third is the SymMap database [30] (https://www.symmap.org/) which builds a large heterogeneous network by combining 19595 herbal ingredients and 4302 target genes related to symptoms [30]. After deleting repeated targets, all the unique targets obtained were considered to be regulated by QUE.

### 2.2. Obtaining Genes Related to DN and Podocyte Injury

Genes associated with DN were retrieved from five comprehensive databases, including the Online Mendelian Inheritance in Man database [31] (OMIM, https://www.omim.org/), DrugBank database [32] (https://www.drugbank.ca/), the Kyoto Encyclopedia of Genes and Genomes Pathway Database [33] (KEGG, https://www.kegg.jp/), and Therapeutic Target Database [34], (TTD, https://db.idrblab.net/ttd/) with the keyword “diabetic nephropathy,” as well as GeneCards database [35] (https://www.genecards.org/), with the keyword “[all] (diabetic nephropathy) and [all] (Homo sapiens).”

Genes related to podocyte injury were searched from four databases: OMIM and DigSee database [36] with the keyword “Podocyte injury” (https://210.107.182.61/digseeOld/), GeneCards database with the keyword “[all] (podocyte injury) and [all] (Homo sapiens),” and Gene Expression Omnibus (GEO) database [37] with the keyword “(Podocyte injury) AND “Homo sapiens”[porgn: txid9606].” From the GEO database, a human gene expression data series (GSE51834) [38] titled “Indoxyl sulfate, a uremic toxin and aryl-hydrocarbon receptor ligand, mediates progressive glomerular disease by damaging podocytes” published in 2014, was selected to explore differential genes (DEGs) of podocyte injury. There was a series matrix file that included three podocyte injury samples and three control samples in this series. The DEGs were gathered by comparing these two types of samples with fold change (FC) of genes expression (|logFC| ≥ 1) and false discovery rate (*P* < 0.05) using the Limma package [39] of the R project software.

### 2.3. Constructing Protein-Protein Interaction (PPI) of Mapping Targets and Identifying Candidate Targets

QUE-associated targets, podocyte injury-related genes, and DN-associated genes were subjected to intersection analysis to identify the mapping targets that were considered to be highly relevant to QUE protecting against podocyte injury in DN. The “protein-protein interaction (PPI)” topological network of the mapping targets was constructed using the STRING database [40] (https://string-db.org) using Cytoscape 3.71 [41]. The nodes of this network represent proteins, and the edges represent the interactions between the two proteins. The targets having interactions with a probabilistic association confidence a score ≥0.4 were identified candidate targets. The network topology parameters, including the “degree” of targets in the PPI network were analyzed using the Network Analyzer plug-in of Cytoscape. The top three targets with the highest “degree” values were defined as three key targets for QUE protecting against podocyte injury in DN.

### 2.4. Enrichment Analysis of GO Term and KEGG for Candidate Targets using ClueGO and R Project, Respectively

The candidate targets were imported into the ClueGO plug-in [42] of Cytoscape and R project for Gene Ontology (GO) term and KEGG enrichment analysis, respectively, to decipher the molecular mechanisms of QUE protecting against podocyte injury. The results gathered from above two enrichment software were further analyzed and compared, and the most reliable signaling pathway (the largest percentage or the lowest *P* value) was considered to be the major pathway for QUE protecting against podocyte injury in DN.

GO terms describe the biological function of genes through three semantic terms, namely, biological process (BP), cellular component (CC), and molecular function (MF) [43]. KEGG consists of artificially annotated metabolic pathways and defines the complex interrelationship between genes and metabolites [33]. R project software has been widely used in network pharmacology studies for screening of DEGs, enrichment, and annotation analysis [37, 44].

### 2.5. Docking QUE with Key Targets

The interaction between QUE (ligand) and key targets (receptors) were evaluated using Autodocktools-1.5.6 [45] and visualized through PyMOL [46], being able to calculate and analyze the binding affinity and binding energy. The structure of QUE (as a mol2 file) and the targets (as a PDB file) were downloaded from PubChem (https://pubchem.ncbi.nlm.nih.gov/) and the Protein Data Bank database (PDB) (https://www.rcsb.org/pages/contactus), respectively.

## 3. Result

### 3.1. QUE-Associated Targets

A total of 355 targets of QUE (Supplementary Table 1) were obtained from TCMSP (148 targets), SwissTargetPrediction (99 targets), and SymMap (108 targets) databases, and 247 unique targets of QUE were gathered after deleting 108 repeated targets. And, there were six targets (AKT1, TOP1, PARP1, MMP9, MMP3, and MMP2) recorded in those three databases.

### 3.2. 3387 Genes Associated with DN and 816 Genes Related to Podocyte Injury

A total of 4895 human genes (Supplementary Table 2) associated with DN were identified from those five databases, and 3387 unique genes of DN were obtained after deleting 1508 duplications.

848 human genes (Supplementary Table 3) related to podocyte injury were identified, of which 316 were DEGs (130 upregulated genes, including TNFAIP6, TNFAIP3, and VEGFA and 186 downregulated genes, including TNFRSF19 and COL1A1) (Figure 2(a)), 532 of which were obtained from the OMIM (191 genes), GeneCards (339 genes), and DigSee (2 genes) databases. Totally 816 unique genes of podocyte injury were gathered after deleting 32 duplications.

### 3.3. 41 Candidate Targets from PPI Network Analysis of 42 Mapping Targets Related to QUE, DN, and Podocyte Injury

Through intersection analysis QUE-associated targets, DN-associated genes and podocyte injury-related genes, 42 mapping targets (Figure 2(b), Supplementary Table 4) were identified closely related to QUE protecting against podocyte injury in DN.

In total, 41 candidate targets (Figure 3(a), Supplementary Table 5), including 13 DEGs (2 downregulated and 11 upregulated genes (Figure 3(b)) were identified through the PPI network of 42 mapping targets. The PPI network contained 41 nodes, 340 edges with an average “degree” value (the mean number of connections per node) of 16.585. There were 21 candidate targets with a “degree” value ≥average “degree” (Table 1), and the top three targets TNF, VEGFA, and AKT1 ranked by degree were identified as the key targets of protecting against podocyte injury in DN.

### 3.4. Results of Enrichment Analysis about Candidate Targets

A total of five signaling pathways (Figure 4(a)) and 10 biological functions (*P* < 0.05, Figure 4(b)) involving in QUE protecting against podocyte injury were obtained via ClueGO, respectively. Detailed information of ClueGO enrichment results is listed in Table 2. 118 signaling pathways (*P* < 0.05, Supplementary Table 6) and 52 biological functions (*P* < 0.05, Supplementary Table 7) were obtained via R project, respectively. The top 20 signaling pathways with low *P* values are shown in Figure 5.

The top pathway obtained in ClueGO (accounting for 94.44%) and R project (*P*=3.655 × 10^−19^; count = 15) both was the AGE-RAGE signaling pathway in diabetic complications that was also identified as the major signaling pathway of QUE protecting against podocyte injury in DN. Oxidoreductase activity, antioxidant activity, and peroxidase activity from R project were consistent with the regulation of reactive oxygen metabolism (36.92%) from ClueGO [47], and growth factors, cytokine receptors, and protein phosphatase 2A from R project were consistent with endothelial cell proliferation (26.92%) from ClueGO [48].

### 3.5. Results of Molecular Docking

The molecular docking analysis showed that QUE (ZINC3869685) could easily enter and bind to the key target TNF (2JG9), VEGFA (1MKK), and AKT1 (1UNR) with several interactions, hydrogen bonds, and amino acid residues, shown in Figure 6. QUE can form five H-bonds with GLY-201 (2.1), HIS-101 (2.5), SER-207 (2.8), and HIS-101 (2.5 and 1.8) of TNF, eight H-bonds with LEU-66 (2.8), CYS-26 (2.6 and 2.4), GLU-64 (2.4), PHE-47 (2.4), SER-50 (2.5), and SER-24 (2.2 and 3.5) of VEGFA. And, the binding energy of QUE and TNF, VEGFA and AKT1 were −6.35 kJ/mol, −6.75 kJ/mol, and −5.36 kJ/mol, respectively.

## 4. Discussion

The present study shows that QUE would protect against podocyte injury in DN mainly by regulating the major AGE-RAGE signaling pathway and three key targets: TNF mediating the proinflammatory, VEGF promoting vascular permeability and proliferation, and AKT1 participating in apoptosis. Furthermore, QUE, having the five hydroxy groups (placed at the 3-, 3′-, 4′-, 5- and 7-positions), should have suitable binding sites with three key targets and interacts with amino acid residues of targets through multiple hydrogen bonding and Van der Waals using molecular docking analysis.

QUE regulates the oxidative stress-associated AGE-RAGE signaling pathway to protect against podocyte injury in DN. It is known that the binding of AGEs to the receptor RAGE can induce oxidative stress and inflammation, eliciting podocyte injuries [49, 50]. Encouragingly, Li et al. validated that QUE can reduce the production of AGEs by trapping 50.5% of glyoxal and 80.1% of methylglyoxal which are the crucial reactive dicarbonyl precursors of AGEs [51]. Moreover, QUE decreases the expression of RAGE [52] and increases the expression of superoxide dismutase (SOD) to suppress oxidative stress accelerated by the activated AGE-RAGE pathway, protecting the cell from injury [53]. Additionally, QUE is an antioxidant, it can not only increase the expression of podocyte slit diaphragms and sensitive markers of podocyte nephrin and podocin to the maintenance of the skeletal structure and function of podocytes [23, 54] but also lower the kidney hypertrophy index (KI), blood urea nitrogen (BUN), and blood creatinine (Scr) to improve kidney function in diabetic rats [52]. Therefore, it can be inferred that QUE can prevent podocytes from the stimulation of oxidative stress by inhibiting HG which induced excessive accumulation of AGEs, lowering ROS synthesis. Furthermore, accumulating evidence has also shown there is a close relation between the AGE-RAGE signaling pathway and other complications of diabetes such as diabetic peripheral neuropathy and diabetic retinopathy [55–57]. Therefore, QUE might also have preventive effects on complications of diabetes.

QUE inhibits key targets of TNF mediating the proinflammatory and regulates VEGF promoting vascular permeability and AKT mediating apoptosis to protect podocytes from injury in DN. Experiments in the streptozocin-induced diabetic rat have demonstrated that the inflammatory cytokine of TNF-*α*, a member of the TNF receptors superfamily, is an intermediate factor for excessive ROS-induced podocyte injury and apoptosis [58–60]. Moreover, TNF-*α* plays a predictive role in DN, attributing to its involvement in the onset and progression of DN [61]. Encouragingly, QUE has been proven to decrease the renal TNF-*α* and ROS synthesis [62] induced by high homocysteine (Hcy) [63] which is an independent risk factor for DN [64]. High Hcy can also directly cause podocyte injury, with subsequent progression of glomerular permeability induced by oxidative stress [64, 65], and can affect the function of renal endothelium and mesangial cells during the progression of DN [66, 67]. While, as DN progresses further, abnormal elevation of Hcy directly damages vascular endothelial cells and aggravates microalbuminuria and ultimately forms a vicious circle between DN and Hcy [65, 68]. Interestingly, QUE can also reduce the level of Hcy and increase the level of the Hcy's metabolite, taurine, an antioxidant that has been demonstrated to improve glomerular sclerosis and attenuate the progression of DN in mice [69, 70]. Metabolomic studies have consistently shown that QUE increases the level of taurine in mice serum and urine [70, 71]. Treatment with taurine significantly downregulates the protein levels of podocyte homeostasis regulator and consequently the reduction of glucose-induced podocytes injuries in DN mice model [72]. Furthermore, high Hcy-induced endothelial cell apoptosis is commonly associated with increased VEGF [73]. VEGF is the important mediator in endothelial cell proliferation and glomerular mesangial proliferation at the end-stage of DN [74]. It is regulated by candidate target ERK1/2 (also known as MAPK1, degree = 24) and key target AKT (degree = 31), and the excessive production of VEGF subtype A (VEGFA), resulting from the interaction of AGEs and RAGE, is a novel risk factor in the pathogenesis of the endstage renal disease [55, 75]. But excessive inhibition of VEGF causes glomerular injury with prominent podocyte injury [76, 77]. So, it would be speculated that the therapeutic index of VEGF for podocyte injury is narrow, which is in line with the statements of Oe et al. [78]. Interestingly, QUE can moderately regulate the expressions of VEGFA and alleviate podocyte injury and kidney function in diabetic rats [23]. Hence, QUE is a new appropriate product that targeted VEGFA to ameliorate podocyte injury. The phosphorylation of another key target AKT can significantly prevent from podocyte apoptosis, foot process shrinkage, and renin loss [78]. However, the levels of phospho-Akt are downregulated by long-term HG, causing the increased activation of p38 MAPK and renal proximal tubule cell apoptosis [79]. Noteworthily, QUE can increase the phosphorylation of AKT to promote the synthesis of liver glycogen with lowering blood sugar and regulate the downstream proteins of AKT to facilitate lipid metabolism [80]. Thus, it can be assumed that QUE promotes glycogen synthesis via AKT phosphorylation to prevent podocytes from injury. In addition, QUE inhibits the expression of candidate target TP53 being a key regulator of p53 apoptotic signaling pathways which are involved in podocyte senescence and apoptosis [80, 81], and the downstream signaling pathways of TP53, such as NF-kB signaling pathways, that participate in HG-induced podocyte injury [82, 83].

Moreover, this study also indicates that QUE protects against podocytes injury having relation with autophagy from enrichment analysis (*P*=0.0048 from the R project). Autophagy, which can accelerate the metabolism of ROS induced by HG, significantly accelerates the metabolism of ROS and inhibits the activation of VEGF, showing its importance to maintain the postmitotic podocytes cells [84, 85]. More and more researches prove that QUE can suppress ROS synthesis through induction of autophagy to cure liver fibrosis and CVD [86–88]. Additionally, QUE can significantly upregulate autophagy by suppressing oxidative stress and downregulating TNF-*α* and AKT and ameliorating doxorubicin-induced podocyte injury in rats [89, 90]. Thus, it can be hypothesized that QUE may act on autophagy associated with the reduction of ROS to participate in the protection of podocytes injury [91, 92].

Although it has been confirmed in different experimental models that QUE regulates key targets at TNF, VEGFA, and AKT1, as well as the AGE-RAGE signaling pathway to protect against podocyte injury. In this article, the findings suggest that the multipronged therapeutic effect of QUE on podocyte injury, attributing to its synergistic effects on these multiple targets. However, further experimental studies will be needed to verify it.

## 5. Conclusion

This study reveals that QUE can reduce the inflammatory response (TNF and IL6), inhibit endothelial cell proliferation (VEGFA) and apoptosis of podocytes (AKT1 and TP53), and suppress the AGE-induced oxidative stress by regulating the AGE-RAGE signaling pathway activated by HG to protect against podocytes injury in DN (Figure 7). This study provides a scientific basis for developing QUE as a potential natural medicine for the treatment of DN.

## Figures and Tables

**Figure 1:** Flow chart of network pharmacology method used in this study.

**Figure 2:** (a) Volcano map of 316 differential genes of podocyte injury. The 130 upregulated genes are presented in red, whereas 186 downregulated genes are presented in green. (b) Venn diagram and PPI network showed the 42 mapping targets of QUE protects against podocytes injury in DN.

**Figure 3:** (a) 41 candidate targets obtained from network of “protein-protein” interaction (PPI), including three key targets TNF (degree = 34), VEGFA (degree = 33), and AKT1 (degree = 31). The color of the nodes is shown in a gradient from to red to transparent according to the degree value. (b) 13 DEGs contained in 41 candidate targets, the red bars represents11 upregulated genes (log C 1), and the green bars represents 2 upregulated genes (log FC < −1).

**Figure 4:** The enrichment results of KEGG (a) and GO terms analysis (b) for the 41 candidate targets via ClueGO. The AGE-RAGE signaling pathway is the most reliable pathway in ClueGO (94.44%), regulation of reactive oxygen metabolism (36.92%) and endothelial cell proliferation (26.92%) are top two reliable biological functions.

**Figure 5:** Enrichment results of KEGG (a) and ClueGO (b) from R project. The AGE-RAGE signaling pathway (*P*=3.655 × 10^−19^; count = 15) is also the most reliable pathway R project.

**Figure 6:** 3D molecular binding model of QUE to key targets TNF, VEGFA, and AKT1. Three key targets are represented as light blue flat strips, and amino acid residues of key targets are represented as colored sticks and QUE is represented as the yellow stick. The yellow dashed lines demarcate hydrogen bonds, and the interaction distances are indicated next to the bonds.

**Figure 7:** Effects of QUE protecting against podocytes injury in DN via key targets TNF, VEGFA, and AKT1 in AGE-RAGE signaling pathways.

**Table 1:** 21 candidate targets with a degree greater than average.

Target	Uniprot ID	Description	Degree
TNF	P01375	Tumor necrosis factor	34
VEGFA	P15692	Vascular endothelial growth factor	33
AKT1	P31749	AKT serine/threonine kinase 1	31
TP53	P04637	Tumor protein p53	29
PTGS2	P35354	Prostaglandin G/H synthase 2	28
CXCL8	Q9UI36	C-X-C motif chemokine ligand 8	28
JUN	P05412	Jun proto-oncogene,	27
IL10	P22301	Interleukin-10	25
IL1B	P01584	Interleukin-1 beta	24
MAPK1	P10911	Mitogen-activated protein kinase 1	24
CCND1	P24864	Cyclin D1	22
HMOX1	P09601	Heme oxygenase 1	21
STAT1	P42224	Signal transducer and activator of transcription 1-alpha/beta	21
APP	P05067	Amyloid beta precursor protein	21
VEGF2	P35968	Vascular endothelial growth factor receptor 2	20
PTEN	P60484	Phosphatase and tensin homolog	20
CRP	P02741	C-reactive protein	20
SELE	Q5TI75	Selectin E	18
F2	P16930	Coagulation factor II, thrombin	17
HIF1A	P01892	Hypoxia inducible factor 1 subunit alpha	17
SOD1	P00441	Superoxide dismutase 1	17

**Table 2:** KEGG (*A*) and GO (B) term enrichment results from ClueGO.

ID	Description	Percentage	Count
A			
KEGG: 04933	AGE-RAGE signaling pathway in diabetic complications	94.44%	36
KEGG: 05418	Fluid shear stress and atherosclerosis	1.39%	15
KEGG: 04610	Complement and coagulation cascades	1.39%	4
KEGG: 05014	Amyotrophic lateral sclerosis (ALS)	1.39%	3
KEGG: 04923	Regulation of lipolysis in adipocytes	1.39%	3

B			
GO: 1903409	Reactive oxygen species biosynthetic process	36.92%	18
GO: 0001937	Positive regulation of endothelial cell proliferation	26.92%	24
GO: 0048662	Positive regulation of smooth muscle cell proliferation	12.31%	20
GO: 0001936	Regulation of endothelial cell proliferation	8.84%	17
GO: 2000377	Regulation of reactive oxygen species metabolic process	5.34%	31
GO: 0014074	Response to purine-containing compound	5.34%	17
GO: 0045766	Positive regulation of angiogenesis	2%	17
GO: 0007589	Body fluid secretion	2%	6
GO: 0042730	Fibrinolysis	2%	5
GO: 0001937	Negative regulation of endothelial cell proliferation	2%	3

## Data Availability

The data of this research is obtained through authoritative online databases and software analysis and can be acquired from the Supplementary Materials uploaded with this article.

## Supplementary Materials

Supplementary Materials Supplementary Table 1: 355 targets of QUE. Supplementary Table 2: 4895 human genes related to DN. Supplementary Table 3: 848 human genes associated with podocyte injury. Supplementary Table 4: 42 mapping targets. Supplementary Table 5: specific analytical parameters of 41 candidate targets. Supplementary Table 6: 118 signaling pathways from R project. Supplementary Table 7: 52 biological functions from R project.
